The article "How does multidimensional R&D investment affect green innovation? Evidence from China" was retracted in 2025. Reasons: an official misconduct investigation; compromised peer review; a compromised editor; unreliable results or conclusions.

# How does multidimensional R&D investment affect green innovation? Evidence from China

**DOI:** 10.3389/fpsyg.2022.947108

**Published:** 2022-08-24

**Authors:** Yang Shi, Can Yang

**Affiliations:** ^1^School of MBA, Shandong University of Finance and Economics, Jinan, China; ^2^SINOTRUK Finance Co., Ltd., Jinan, China

**Keywords:** system quality, R&D investment, green innovation ability, threshold effect, China

## Abstract

Under the background of green development, multidimensional R&D investment and institutional quality have injected strong power into green innovation. Based on China's provincial panel data from 2009 to 2018, this study examines the threshold effect of R&D and R&D personnel input on China's green innovation capability from three perspectives, namely, political institutional quality, economic institutional quality, and legal institutional quality. The core study results show that the influence of R&D on China's green innovation capability has an obvious double-threshold effect based on institutional quality. This study expands the research on the influencing factors of green innovation and the influence effect of multidimensional R&D investment and provides a theoretical basis for regional green innovation management. In addition, the research results of this study provide a reference for accurately formulating regional green innovation capability promotion strategies.

## Introduction

Since the reform and opening up, China's economy has grown rapidly and the level of national welfare has practically improved, creating a “Chinese miracle.” Behind the high growth, the extensive development model has made China pay a heavy price in terms of resources and the environment, and the ecological and environmental problems are prominent (Hao et al., 2022). China's economy is in urgent need of transformation, from the pursuit of quantity expansion to the pursuit of quality and efficiency. Accelerating green technology innovation and improving green innovation ability is the breakthrough point of economic green transformation (Sun et al., 2020a,b,c), and also important support for promoting China's high-quality, sustainable, and green development. In the endogenous economic growth model, technological progress is the decisive factor in the economic growth (Furman et al., 2002; Lucas, 2015). China's “14th Five-Year Plan” points out that it is necessary to “vigorously develop the green economy” and “build a green technology innovation system.” It is clear that green innovation is the first driving force to drive green development and the strategic support to realize economic development and environmental protection. Therefore, with the increasingly prominent environmental problems and the strategic position of green innovation capability, we should constantly explore the promotion path of green innovation in theoretical and empirical analysis.

With the continuous improvement of the national innovation system and the continuous advancement of industrialization, the national R&D investment and the R&D capability of enterprises play a key role in enhancing the green innovation capability of high-tech enterprises in China (Wu et al., 2021). On the one hand, the state's support for enterprises' green innovation continues to increase, prompting enterprises to continuously carry out green innovation (Berger et al., 2019; Tang et al., 2022). On the other hand, the state's financial support for green innovation has reached record highs, which makes enterprises' enthusiasm and consciousness to participate in green innovation constantly improve, and they tend to introduce increasing technology and R&D talents to enhance their R&D and innovation capabilities, so as to continuously improve the innovation performance of enterprises and further enhance the innovation awareness and innovation capability of the whole country (Leung, 2015). Besides, institutional quality also has an important impact on innovation (Sun et al., 2021b). Actually, it is necessary for the increase of R&D investment to promote the improvement of green innovation capability (Ren et al., 2021; Wang et al., 2022). What are the specific conditions for R&D investment to improve China's green innovation capability? What factors affect the direction and degree of technology spillover effects of R&D investment and then make China's green innovation capability appear heterogeneous? Based on the institutional quality, it is of great decision-making value for top-level design in environmental policy and regional green innovation to investigate the non-linear influence of R&D investment on green technology innovation.

The possible marginal contributions of this study are as follows. First, on the basis of integrating the existing theories, this study brings institutional quality, R&D investment, and green innovation into a unified research framework, which broadening scope of green innovation research and forming a conclusion close to the objective reality. Second, empirically, this study analyzes the non-linear impact of multidimensional R&D investment on green innovation using the threshold model, which can more accurately analyze the path of R&D investment on China's green innovation capability. Third, in the practical sense, based on the quality of the economic system, political system, and legal system, this study confirms the effect of R&D investment in the process of green innovation and provides a practical thinking direction for the improvement of green innovation capability.

## Literature review

Some scholars have studied the influence of R&D investment on innovation (Ahmad and Zheng, 2022; Wan et al., 2022; Zhang and Mohnen, 2022), and the influence mechanism of technology investment on national innovation ability has been revealed (Sun et al., 2021a,b; Li et al., 2022). R&D is the core element of innovation, which will accumulate human capital and knowledge stock and enhance the capacity of innovation (Irfan et al., 2021; Boeing et al., 2022). Pang et al. (2014) and Zhou and Zhu (2017) based on the data of 426 innovative enterprises and macro data in China, respectively, confirmed that R&D investment is a booster for innovation performance using the government-enterprise correlation theory and econometric model. Ginarte and Park (1997) found that advanced scientific and technological equipment and means play an important role in promoting major fundamental innovation based on the study of major innovation cases in history. Gooch et al. (2017) studied the R&D investment and performance of about 1,000 large manufacturing companies in the United States from 1957 to 1977, and the R&D investment has always been an important contribution to the production efficiency of enterprises. According to the data of American pharmaceutical companies from 1950 to 2008, it is further found that the umbilical link between the acquisition of enterprise patents in the pharmaceutical industry and the continuous R&D expenditure, which indicates that the scientific research investment of enterprises not only improves the production efficiency but also greatly improves the innovation ability of enterprises (Kunapatarawong and Martínez-Ros, 2016). Innovation and technology policy can serve innovative enterprises from the perspective of resources and dynamic evolution and further enhance their ability to innovate (Berger et al., 2019).

In addition to the technological investment of enterprises, the government's special funds for technology also inject a “stimulant” into innovation (Wen et al., 2022). Diversified financial special investment has guided all sectors of society to pay attention to and support the basic research layout, and the technological innovation governance system has been improved (Wu et al., 2017; Irfan et al., 2021). Wu et al. (2017) using the local government behavior function, starting from the government assessment mechanism and fiscal and tax incentive structure and using the econometric method, revealed that investment has a sustained two-way promoting effect on the original innovation capability. Mei and Luo (2020) found that financial subsidies can encourage private enterprises, especially high-tech enterprises, to create higher innovation performance using the special database of high-tech enterprises at Northwest A&F University. The contribution of R&D input factors to patent production in China is measured using the Douglas production function and the Solow residual method. It is further shown that the contribution of R&D expenditure is more than three times that of R&D personnel's full-time equivalent (Weng and Wang, 2011). Starting from the structure of science and technology investment, some studies discuss the effects of government funding, financial market financing, and enterprise self-financing on green innovation capability (Yang et al., 2021; Sun and Razzaq, 2022).

In the research of related fields, scholars mostly focus on pollution permits systems (Ren et al., 2022a,b) and corporate social responsibility disclosure (Hong et al., 2020), and financial resource allocation (Jia et al., 2021; Su et al., 2021; Bhatnagar et al., 2022; Khan et al., 2022), environmental regulation (Xu et al., 2022), financial technology (Yao et al., 2021), and other perspectives have studied the influencing factors of green innovation. Few scholars have paid attention to the institutional environment and green innovation capability of R&D investment. This study fills this gap. Most related studies are limited to linear analysis. However, due to the huge heterogeneity of green R&D in China, linear research cannot describe the relationship in detail. Different from previous studies, this study adopts a new perspective of institutional quality, which has been ignored in the previous literature, and subdivides institutional quality into political, economic, and legal system quality. The threshold panel model is applied to analyze and clarify the influence and mechanism of institutional quality in the effect of R&D investment on green innovation capability.

## Research hypothesis and empirical design

### Research hypothesis

In 1930s, Wassily W.·Leortief put forward the input–output theory, which provided a practical economic analysis method. The theory was mostly used for macro-phenomenon analysis and then extended to microfield (Hewings et al., 1988). This theory provides a theoretical basis for this study to examine the influence of R&D input on green innovation. Specifically, the process from R&D investment to green innovation is essentially an input-output process. R&D personnel and R&D funds are input elements, and green innovation is the resultant output of the innovation process (Fan et al., 2021). The input of R&D personnel can provide the intellectual foundation for green innovation, and talents are the core driving force of green innovation and play a key role in the process of green development (Li et al., 2019). On the one hand, the skills, ideas, and creativity of R&D personnel can transform R&D resources into innovative achievements. On the other hand, R&D talents have the characteristics of wide regional distribution and high industry penetration density. Increasing the input of R&D personnel can give full play to the knowledge spillover effect, that is, through the communication between R&D personnel, the innovation output can be highly efficient (Sánchez-Sellero and Bataineh, 2021). In addition, the input of R&D funds is the basic guarantee of green innovation output (Bai et al., 2019), and it is the prerequisite for purchasing production equipment and recruiting high-tech talents. Therefore, this study puts forward the following research hypotheses:

H1: Multidimensional R&D investment can promote green innovation.

Green innovation is inseparable from institutional quality (Sun et al., 2019). Whether the institution is effective is an important factor that affects the smooth development of green innovation R&D activities (Yuan et al., 2022). For regions with high system quality, policy implementation is more efficient, government governance ability is stronger, enterprise innovation risk is lower, and intellectual property protection will be stronger. Therefore, enterprises have more initiative and enthusiasm in carrying out green innovation activities (Arshed et al., 2022). Accordingly, this study puts forward the following research hypotheses:

H2: The influence of R&D on green innovation is influenced by institutional quality.

### Empirical design

According to previous studies, it is also assumed that the green innovation capability will be influenced by factors such as economic development level, national economic policy regulation, human capital, foreign direct investment, and foreign direct investment (Swart et al., 2014; Jones et al., 2017). To further test hypothesis H2, under different institutional quality, the impact of R&D input on green innovation may not be a simple linear relationship but a threshold effect of institutional quality. Therefore, referring to Hansen (1999), Wu et al. (2019), and Fang et al. (2022), this paper uses panel threshold model to test the non-linear influence of multidimensional R&D input on green innovation. Compared with other models that test the interval effect, the panel threshold model has the advantage of reducing the errors caused by the subjectivity of artificial interval division.


(1) $$\begin{array}{l} lncreate_{it}=\beta_{0}+\beta_{1}lncore_{it}I\left(q_{it}≦M\right)\\ \;\begin{array}{l} +\;\beta_{2}lncore_{it}I\left(q_{it}>M\right)\\ +\;\beta_{n}x_{it}+\alpha_{i}+e_{it} \end{array} \end{array}$$

where *create*_*it*_ means green innovation, and *core*_*it*_ represents core explanatory variables, including R&D capital investment and R&D personnel investment. The model constructed with different core explanatory variables is similar to formula (1), and only the core explanatory variables need to be replaced separately, so it is unnecessary to repeat; *x*_*it*_ represents control variables, including economic development level, national economic policy regulation, human capital, and FDI; *e*_*it*_ represents a random perturbation term; *q*_*it*_ indicates the threshold variables, including the system quality of the political, economic, and legal; (·) is a characteristic function; *M* is the particular threshold value; α_*i*_ means area fixed effect; Ln is logarithm; and β_0_ and β_1_, β_2_, …, β_*n*_ are constants and parameters to be estimated.

### Explanation of variables

1. Explained variables
  Green innovation ability (*Create*). Following previous studies (Tang et al., 2021), the number of provincial green patent applications is used. The data in each province are from the China Intellectual Property Office.
2. Core explanatory variables
  R&D capital investment (*Rci*) is expressed by the ratio of regional R&D spending and GDP. The full-time equivalent of R&D personnel (10,000 people) is used as a proxy variable for regional R&D personnel investment (*Rpi*).
3. Threshold variable
  Political system quality (*politic*). Due to the complexity of *politic*, regional corruption is regarded as the proxy variable of *politic* for simplicity, specifically the number of crimes filed per 10,000 civil servants. In this study, corruption is defined as “public power being used to pursue personal interests in violation of rules.”

Economic system quality (*economic*). Based on previous studies, the *economic is* represented by China's marketization index, and the data are from the China's marketization index. Among them, 2010–2014 market-oriented index data are missing. Based on Fan Gang's 1997–2009 market index total score data, the heterodyne values are padded with regression.

Legal system quality (*protect*). Intellectual property protection is applied to represent *protect*. For *protect*, the index composition is shown in Table 1. The Ginarte-Park method is used for weight setting.

4. Control variables
  FDI in different provinces is the actual use of foreign direct investment (million US dollars). OFDI is the net non-financial foreign direct investment (US$10,000) of China's provinces over the years. The data come from the Wind database, Human capital (Hum). Referring to the previous studies, the weighted average of the educational years of the population over 6 years old is used. State economic regulation and control (EP): EP is measured by the ratio of the fixed assets investment amount of the state-owned and its holding enterprises in each region to the total fixed assets investment in the region. Table 2 shows the description of the variables.

**Table 1:** Legal system quality index system.

**Primary indicators**	**Secondary indicators**	**Index description**
Judicial protection level	Number of district lawyers	Number of district lawyers/total district population
	Regional population	
Administrative protection capacity	Regional patent authorization	(Number of infringement cases closed + number of other patents closed + number of cases of counterfeiting others)/amount of patent authorization
	Annual number of patent infringement cases in the region	
	Number of other patent cases	
	Number of cases of counterfeiting others' patents	
Economic development level	Regional real GDP	Real GDP/regional population
	Regional population	
Education level	Proportion of college students and above	Junior college * 16 + senior high school * 12 + junior high school * 9 + primary school * 6
	Proportion of high school culture	
	Proportion of junior high school culture	
	Proportion of primary schools	

The data are from China Statistical Yearbook, China Lawyer Yearbook, and China Intellectual Property Protection Bureau.

**Table 2:** Statistical description of variables.

**Variable name**	**Symbol**	**Sample**	**Mean**	**S.d**	**Min**	**Max**
Green innovation ability	Create	300	7459.882	21888.58	0	207663.3
Number of patent applications	Patent	300	2616.637	6772.378	0	58,119
Foreign direct investment	FDI	300	626247.3	998450.4	2044	13,100,000
Foreign direct investment	OFDI	300	63707	118559.6	0	1,089,671
Foreign trade	Trade	300	9685678	1.76E+07	41330.7	109,000,000
R&D capital investment	Rci	300	0.847091	0.404499	0.000795	2.831642
R&D personnel input	Rpi	300	82696.23	91790.07	1209	511,718
Quality of economic system	Economic	300	7.835733	2.254093	3.09	14.45
Quality of political system	Politic	300	3.483683	1.130756	1.371849	8.862232
Quality of legal system	Protect	300	1.600317	0.834688	0.695768	5.210585

## Measurement results and empirical analysis

### Threshold model examine

Under the hypothesis of single, double, and triple threshold, bootstraps are adopted to test the threshold effects of *politic*, economic, and *protect* with *Rci* and *Rpi* as core explanatory variables. The results show that (see Table 3) when *Rci* and *Rpi* are the core explanatory variables, taking *politic*, economic, and *protect* as threshold variables, the existence of a double threshold is confirmed. The corresponding threshold estimates and confidence intervals are shown in Table 4.

**Table 3:** Threshold effect self-sampling inspection.

**Core variables**	**Threshold variable**	**Model**	***F*-value**	***P*-value**	**BS times**	**1%**	**5%**	**10%**
Rci	Politic	Single threshold	21.773**	0.017	300	24.823	12.595	8.959
		Double threshold	0.410*	0.067	300	3.380	0.537	−0.786
		Triple threshold	1.581**	0.017	300	2.456	−9.570	−1.981
	Economic	Single threshold	15.634**	0.027	300	22.98	10.965	7.688
		Double threshold	22.833*	0.060	300	36.324	24.137	18.309
		Triple threshold	0.000	0.697	300	0.000	0.000	0.000
	Protect	Single threshold	11.194	0.207	300	33.097	23.426	17.544
		Double threshold	39.067***	0.000	300	17.486	8.399	4.502
		Triple threshold	0.000	0.437	300	0.000	0.000	0.000
Rpi	Politic	Single threshold	10.591**	0.200	300	14.185	7.158	5.385
		Double threshold	26.598***	0.000	300	7.290	3.282	2.391
		Triple threshold	0.000	0.813	300	0.000	0.000	0.000
	Economic	Single threshold	10.167*	0.063	300	21.029	11.948	8.243
		Double threshold	20.467**	0.020	300	23.575	13.818	8.243
		Triple threshold	0.000	0.623	300	0.000	0.000	0.000
	Protect	Single threshold	10.604*	0.070	300	20.524	12.761	8.482
		Double threshold	16.290***	0.003	300	10.151	5.960	3.724
		Triple threshold	0.000	0.437	300	0.000	0.000	0.000

***, **, and * are significant at 1%, 5%, and 10% levels, respectively. The p-value and the bootstrap is 300 times.

**Table 4:** Threshold estimates and their confidence intervals.

**Core variables explain**	**Threshold variable**	**Model**	**Threshold estimates**	**95% confidence interval**
Rci	Political system	Double threshold model	2.621	[2.499, 2.621]
			2.703	[2.673, 2.978]
	Economic system	Double threshold model	8.960	[7.170, 10.020]
			7.440	[4.400, 12.710]
	Legal system	Double threshold model	0.870	[0.869, 0.891]
			2.794	[0.909, 3.214]
Rpi	Political system	Double threshold model	2.634	[2.593, 2.662]
			2.227	[2.071, 2.247]
	Economic system	Double threshold model	9.380	[4.400, 10.020]
			5.040	[4.400, 8.780]
	Legal system	Double threshold model	1.523	[1.364, 1.617]
			0.890	[0.870, 0.898]

### Threshold regression results

(1) The quality of the political system. According to Tables 4, 5, the influence of *Rci* on *Create* has a double threshold effect based on the quality of the political system (*politic*). When the level of regional corruption (*Cor*) is low, less than the first interval value of 2.621, the quality of the political system is relatively high. The key coefficient is 1.851; when the level of *rent-seeking* or regional corruption increases (*Cor*), the results show that the quality of the political system is further reduced, and the promotion effect of Rci on *Create* is significantly reduced, which is 1.683; when the level of regional corruption continues to cross 2.703, the quality of the political system is further reduced, but the promotion effect is reduced to 1.607. In brief, with the improvement of political system quality, R&D plays an increasingly important role in promoting green innovation ability. The reason may be that political corruption will make the financial investment in education and R&D innovation insufficient, and a large number of talented people in scientific research and innovation will be lost (Xu and Yano, 2017). Therefore, institutional factors are considered as the decisive factors in promoting green innovation. With the improvement of political system quality, that is, the reduction of regional corruption, the scientific research activities with green innovation as the carrier have been promoted, and the revolutionary transformation of traditional production methods and technical levels has been promoted, thus enhancing the regional green innovation capability (Lee et al., 2020).
(2) The quality of the economic system. When the *economic* is lower than 7.440, the coefficient of *Rci* is 1.388, and the increase of *Rci* is remunerative for *economic*; when the economic system quality is >7.440 and <8.960, the coefficient of *Rci* is 1.967, and the R&D elasticity coefficient increases; when the quality of the economic system is >8.960, the promotion effect of *Rci* increases to 2.491. On the whole, with the improvement of the quality of the economic system, the influence coefficient of R&D on green innovation ability increased from 1.388 to 2.491. The reason is that the continuous improvement of the quality of the economic system is helpful to speed up the construction of a market-oriented green technology innovation system and also to stimulate the enthusiasm of enterprises to develop green technology, thus promoting the regional green innovation capability (Coccia, 2021).
(3) The quality of the legal system. When the quality of legal system is lower than 0.870, the coefficient of *Rci* is −1.313, and the increase of R&D investment inhibits the improvement of *Create*. When the value of politic is in [0.870, 2.794], the R&D coefficient is 0.692. When the quality of the legal system is >2.794, the promotion effect increases to 1.465. When the quality of the legal system is in the second range, R&D can promote the regional innovation ability the most. The reason may be that the quality of the legal system is too low, which is not conducive to creating a green innovation environment, such as insufficient protection of intellectual property rights (Anderlini et al., 2013). When the requirements of the legal system are too strict, it will also limit the exertion of innovation vitality. Therefore, moderate legal system quality is the most effective way to improve the green innovation ability.

**Table 5:** Threshold results with *Rci* as an independent variable.

	**(1)**	**(2)**	**(3)**
lnFDI	0.148**	0.365***	0.406***
	(2.14)	(4.58)	(6.00)
lnOFDI	0.178***	0.190***	0.114***
	(6.25)	(6.35)	(3.71)
lnHum	3.943***	1.682***	6.181***
	(5.86)	(2.63)	(7.90)
lnEP	−0.997***	−1.040***	−0.755***
	(−5.02)	(−4.83)	(−3.48)
lnGDP	0.311***	0.242***	0.270***
	(4.40)	(3.39)	(3.53)
*lnRci*·*I* (*Regime* ≤ *C*_1_)	1.851***	1.388***	−1.313**
	(9.92)	(11.82)	(−2.38)
*lnRci*·*I* (*C*_1_<*Regime* ≤ *C*_2_)	1.683***	1.967***	0.692***
	(7.42)	(8.20)	(9.74)
*lnRci*·*I* (*C*_2_<*Regime*)	1.607***	2.491***	1.465**
	(14.75)	(11.46)	(2.41)
Constant term	−9.133***	−6.727***	−15.819***
	(−6.42)	(−4.59)	(−9.62)
*F*-test	224.91***	203.89***	229.17***
	[0.00]	[0.00]	[0.00]
*R* ^2^	0.8691	0.8571	0.871
Number of samples	300	300	300

() refers to t-value, and [] refers to p-value. ***, **, and * are significant at 1%, 5%, and 10% levels, respectively.

Table 6 shows the estimation results of the dual threshold model with Rpi as the core explanatory variable.

(1) The quality of the political system. When the level of *Cor* is small and <2.227, the quality of the political system is relatively high, and the impact of Rpi on Create is 0.984, which is significantly positive; when the degree of Cor increases and the value is in [2.227, 2.634], the promotion effect of *Rpi* is significantly reduced to 0.971; and when the level of *Cor* is increasing, the quality of the political system is further reduced, and the promotion effect of Rpi is reduced to 0.923.
(2) The quality of the economic system. When *economic* is in [0, 5.050], the coefficient of *Rpi* is 0.936, and the increasing *Rpi* promotes *Create*; when the quality of the economic system is >5.040 and <9.380, at this time, the elasticity of Rpi is 0.965; and when the *economic* is >9.380, the promotion effect of *Rpi* on *Create* increases to 0.980.
(3) The quality of the legal system. When the quality of the legal system is lower than 0.890, the coefficient of Rpi is 1.105, and *Rpi* has an improved effect on *Create*. When the quality of the legal system is >0.890 and <1.523, the Rpi elasticity coefficient is 1.465. At this time, *Rpi* is a booster in promoting green innovation ability. When the quality of the legal system is >1.523, the promotion effect decreases to 1.205.

**Table 6:** Threshold results with Rpi as the core explanatory variable.

**Explanatory variables**	**(4)**	**(5)**	**(6)**
lnFDI	0.331***	−0.014	0.108*
	(7.01)	(−0.26)	(1.79)
lnOFDI	0.141***	0.075**	0.051*
	(5.78)	(2.52)	(1.83)
lnHum	4.754***	8.489***	7.351***
	(9.28)	(11.63)	(9.28)
lnEP	−0.723***	−0.800***	−0.534***
	(−3.99)	(−3.6)	(−2.88)
lnGDP	−0.045	−0.037	0.057
	(−0.64)	(−0.46)	(0.65)
*lnRPI*·*I* (*Regime* ≤ *C*_1_)	0.984***	0.936***	1.105***
	(14.68)	(8.04)	(9.42)
*lnRPI*·*I* (*C*_1_<*Regime* ≤ *C*_2_)	0.971***	0.965***	1.142***
	(14.55)	(8.36)	(9.88)
*lnRPI*·*I* (*C*_2_<*Regime*)	0.923***	0.980***	1.205***
	(13.8)	(8.43)	(10.22)
Constant term	−19.520***	−22.586***	−23.839***
	(−20.46)	(−15.62)	(−15.53)
*F*-test	302.61	184.01	213.87
	[0.00]	[0.00]	[0.00]
*R* ^2^	0.898	0.845	0.862
Number of samples	300	300	300

() refers to t-value, and [] refers to p-value. ***, **, and * are significant at 1%, 5%, and 10% levels, respectively.

## Conclusion and policy implications

From the institutional quality dimension of economy, politics, and law, the threshold effects of R&D capital investment and R&D personnel investment on China's green innovation capability are tested using evidence from China. The results show that the influence of R&D on China's green innovation presents the characteristics of dual doorsills of system quality. For political system quality, its positive effect on green innovation decreases with the quality of the political system; in areas with low quality of economic system, the good influence of R&D on green innovation continues to increase as the threshold is continuously crossed; and for legal system quality, with its improvement, the impact of R&D on green innovation gradually changes from negative to positive.

The policy implications for promoting green innovation ability in China are as follows:

First, accelerate the improvement of the political, economic, and legal systems. All regions in China should face up to the existence of constructive contradictions in the system and the deficiencies in the system's construction work and should take appropriate countermeasures to solve the difficulties and problems in the process of advancement, so as to better promote the perfection of laws and regulations. Specifically, to deepen the reform of the economic system, we need to speed up the improvement of the modern market system, handle the relationship between the government and the market, speed up the transformation of the economic development mode, speed up the construction of an innovative country, and promote more efficient, fair, and sustainable economic development. For the construction of a legal system, we should actively promote the modernization of legislation, law enforcement, justice, and law-abiding. For the construction of a political system, all regions should intensify anti-corruption.

Second, for areas with imperfect system construction and low institutional quality, we should improve the construction of the financial market system, improve the local laws and regulations, and speed up the construction of regional economic, political, and legal institutional quality. At the same time, we will increase R&D investment, improve the mechanism of government-oriented and social multichannel investment, and increase support for basic frontier research. For the first echelon whose system quality is still at a low level, we should further improve laws and regulations, encourage patent technology applications through multiple channels, and put the cultivation of strategic emerging industries in an important position so as to make these areas cross the second threshold of institutional quality as soon as possible. For areas already in the second and third echelons, they should seize the institutional leading edge, reasonably guide the distribution of investment, and maximize the green innovation effect of R&D.

This article studies the relationship between multidimensional institutional quality and green innovation ability, which has theoretical and practical significance. The policy implications put forward according to the conclusions can promote the improvement of China's green innovation capability. At the same time, this study has some limitations and prospects. First, this article studies the impact of institutional quality from a macro perspective, and the follow-up study is expected to study the impact of institutional quality on enterprises' green innovation capability from a micro perspective; Second, in practice, the promotion of green innovation ability is a complex and dynamic process. If the dynamic threshold model can be used for further research, it is more reasonable in theory.

## Data availability statement

The raw data supporting the conclusions of this article will be made available by the authors, without undue reservation.

## Author contributions

Both authors listed have made a substantial, direct, and intellectual contribution to the work and approved it for publication.

## Conflict of interest

Author CY was employed by SINOTRUK Finance Co., Ltd. The remaining author declares that the research was conducted in the absence of any commercial or financial relationships that could be construed as a potential conflict of interest.

## Publisher's note

All claims expressed in this article are solely those of the authors and do not necessarily represent those of their affiliated organizations, or those of the publisher, the editors and the reviewers. Any product that may be evaluated in this article, or claim that may be made by its manufacturer, is not guaranteed or endorsed by the publisher.
